# Design of a New Catheter Operating System for the Surgical Robot

**DOI:** 10.1155/2021/8898311

**Published:** 2021-01-28

**Authors:** Xu Ma, Jinpeng Zhou, Xu Zhang, Yang Qi, Xiaochen Huang

**Affiliations:** ^1^Tianjin Key Laboratory for Control Theory & Applications in Complicated Industry Systems, College of Electrical and Electronic Engineering, Tianjin University of Technology, Tianjin, China 300384; ^2^Tianjin Key Laboratory of High Speed Cutting and Precision Machining, School of Mechanical Engineering, Tianjin University of Technology and Education, Tianjin, China 300222

## Abstract

In interventional surgery, the manual operation of the catheter is not accurate. It is necessary to operate the catheter skillfully and effectively to protect the surgeon from radiation injury. The purpose of this paper is to design a new robot catheter operating system, which can help surgeons to complete the operation with high mechanical precision. On the basis of the original mechanical structure—real catheter, the operation information of the main end operator is collected. After the information is collected, the control algorithm of the system is improved, and the BP neural network is combined with the traditional PID controller to adjust the PID control parameters more effectively and intelligently so that the motor can reflect the output of the controller better and faster. The feasibility and superiority of the BP neural network PID controller are verified by simulation experiments.

## 1. Introduction

Vascular interventional surgery can be used not only for preoperative diagnosis but also for practical surgical treatment, which is expected to get more applications in future medical practice. However, the development of new technology needs a lot of basic technology support. In addition, because the operation is carried out in the patient, the real-time status cannot be directly monitored [1]. Often, a doctor with rich operation experience is required to insert the catheter manually. For example, in interventional surgery, the catheter is inserted through the patient's blood vessel. In this process, any small mistake will hurt the patient and cause vascular damage. According to experience, a mature neurosurgeon can achieve a surgical accuracy of about 2 mm. However, the contact force between blood vessels and catheters in the human body cannot be detected. However, if an X-ray camera is used during the operation, the long-term operation will cause radiation damage to patients. Moreover, although doctors wear protective clothing, it is difficult to protect their bodies from radiation in the face of X-ray radiation. In order to overcome these problems, we need a better surgical plan and supporting equipment to help and train doctors. The advantages of a robot assistant system are high control precision and remote control. However, compared with the human hand, there is no robot-assisted system that can meet all the technical requirements of vascular interventional therapy.

In this respect, there are many similar application products and research results on the market. One of the popular products is called the da Vinci robot catheter pushing system [2]. The da Vinci system (see Figure 1) provides doctors with more system stability and greater force support during catheter pushing compared with manual tools and can prevent unnecessary radiation exposure to doctors during more precise operations [2].

The Sensei Xi system (see Figure 2) was certified by the FDA and CE, respectively, in 2007 [3]. The system is used for cardiovascular interventional surgery. Doctors can control the remote catheter robot to push the catheter by manipulating the force feedback device. The end of the catheter is equipped with a force sensor, which can let doctors feel the force of the catheter on the blood vessel wall so as to control the catheter.

The core function of the robot system is the propulsion and navigation of the catheter, as well as the force feedback and perception during the propulsion of the catheter. Beijing University of Aeronautics and Astronautics and Institute of Automation of the Chinese Academy of Sciences have carried out research on the propulsion mechanism and end force feedback of the conduit, but no product has been formed yet [4].

In this study, according to the technical requirements of vascular interventional surgery, we designed a new robotic conduit control system [5]. Compared with the robot system mentioned above, our system has a slave consisting of a two-degrees-of-freedom conduit operation platform and a rotatable platform. The slave end is shown in Figure 3, which can complete the conduit turning and inserting operation. In addition, a newly developed force feedback measuring mechanism is developed from the slave end to measure the near side thrust generated when inserting the catheter and provide force feedback to the main end. The surgical robot system has a main end manipulator, as shown in Figure 4, which is called the surgeon's console. The console uses a real catheter instead of the mechanical handle of the previous generation and uses a force sensor (UNCSR, UNIPULSE, Japan; ±nonlinearity 1.0%), torque sensor (OPT-563B, NMB, Japan; ±nonlinearity 0.01%F.S.), DC motor (AM11HS1008-07, MOONS', Japan; step angle accuracy ± 5%), stepping motor (AR Series, Dongfang Electric Machinery, Japan; step angle 0.0036°), and DSP (Texas Ti, TMS320F28335, America) [6]. The communication determines the position and rotation angle of the conduit operated by the slave and provides force feedback to the console operator [7]. The BP neural network PID control algorithm is used to improve the accuracy and real-time manual control operation in the system.

## 2. Robot Conduit Operating System

The mechanical structure design of the surgical robot system is divided into two parts: the main end and the slave end. The surgeon's console is the main side of the system, and the catheter operating end is the slave end of the system. The design is to maintain the same displacement, speed, and rotation angle between the real catheter and the end catheter console [8]. As a result, surgeons can operate the system smoothly and easily. DSP is used as the control unit of each doctor console and catheter console. The doctor console and catheter console establish an Internet-based communication, and the schematic diagram of display communication is shown in Figure 5. The console at the main end sends the axial displacement and rotation angle of the operator to the operating end of the real catheter. At the same time, the operating end of the conduit sends the force signal back to the main end console. The serial communication adopts the communication mechanism of DSP and master-slave connection. The baud rate is set to 19200 B/s [9].

### 2.1. Main End Console

The surgeon's console is shown in Figure 6, called the surgeon's console. The surgeon's console is the main end console, and the whole system is operated by experienced surgeons. The surgeons use the console to perform the operation and use the real catheter to collect the thrust value of the operator and the displacement value and rotation value of the catheter being pushed. The movable part of the operating end of the catheter keeps the same action as the real catheter of the main end. The real conduit is connected to the sensor through a pulley. A DC motor with an encoder is used to generate force-torque feedback, and the motor is fixed on the pulley.

### 2.2. Slave End Console

Figure 7 shows the slave end console. This part is next to the patient. The conduit is inserted by using this device. This part of the mechanical structure contains two degrees of freedom, one is the frame of axial independent motion, and the other is the rotating motion frame [10]. Two clips are installed in this part of the structure. When the surgeon drives the catheter to move and rotate along the axial direction through the main end console, the catheter is clamped by clamp 1, and the catheter maintains its position. When the conduit is clamped, the conduit driving part can move freely through clamp 2 and insert the conduit.

## 3. Control Algorithm

### 3.1. BP Neural Network PID Control Algorithm Introduction

Figure 8 shows a simple model of neuron operation, called the classic “M-P neuron model” [11]. In this model, neurons receive input signals from *n* other neurons connected by weighting. The total input value received by the neuron will be the threshold value of the neuron. The comparison is then processed by an “activation function” to produce the output of the neuron.

In order to improve the control effect of the traditional PID controller, many intelligent control algorithms are introduced, which are combined with the traditional PID controller to produce good results [12]. As a classical intelligent optimization algorithm, the BP algorithm has the advantages of distributed storage, parallel processing, and self-learning, which makes up for the shortcomings of the traditional PID controller. Therefore, BP and traditional PID control are combined to complement each other and optimize the control effect. The input and output samples are learned by the BP algorithm, and the weight value of the network is adjusted in real time so that the output is optimal. Especially for the servomotor system, the self-learning of the BP neural network comes from three important parameters of the PID controller, which can effectively solve the problem that PID control parameters of the motor are difficult to adjust and that the whole system control cannot solve.

Figure 9 shows the block diagram of the BP neural network PID controller system. It is an organic combination of the traditional PID controller and BP neural network. The detailed analysis of each part is as follows.

#### 3.1.1. BP Neural Network Part

The BP neural network is the core part of the BP neural network PID system [13]. Its main function is to adjust the weight coefficient of neurons through self-learning and adaptive ability of the BP algorithm, then adjust three parameters of the PID controller, and optimize the performance of the whole control system. The output signal of the input layer in the BP neural network corresponds to *K*_p_, *K*_i_, and *K*_d_ of the traditional PID controller. The parameter output is shown in Figure 10.

#### 3.1.2. Traditional PID Part

The BP neural network is only an abstract optimization algorithm, and the actual control of the motor still depends on the traditional PID controller [14]. Therefore, the traditional PID part is an indispensable part of the BP neural network PID system. The specific control of the motor still depends on the closed-loop control of the traditional PID controller, so the speed output of the motor follows the input.

### 3.2. Algorithm Simulation

Taking the axial motion of the vascular intervention robot as an example, the dynamic analysis is carried out. Its axial movement is driven by Maxon ec32. The motor pushes the clamp of the whole clamping conduit to move back and forth, thus driving the conduit to move together. According to Newton's second law, the dynamic model of the axial motion of the intervention robot is established:

(1) $$\begin{array}{c} f\left(t\right)=m\ddot{x}\left(t\right)+c\dot{x}\left(t\right)+kx\left(t\right), \end{array}$$

where *f*(*t*) is the motor driving force, *x*(*t*) is the displacement of this motion, $\dot{x}\left(t\right)$ is the motion velocity, and $\ddot{x}\left(t\right)$ is the motion acceleration, and formula (1) illustrates the relationship between motor drive force and output displacements.

If *x*_1_(*t*) = *x*(*t*) and $x_{2}\left(t\right)=\dot{x}\left(t\right)$, then

(2) $$\begin{array}{c} \left\{\begin{array}{c} \dot{x}\left(t\right)=AX\left(t\right)+Bu\left(t\right),\\ y\left(t\right)=CX\left(t\right), \end{array}\right. \end{array}$$

where $X\left(t\right)=\left[\begin{array}{c} x_{1}\left(t\right)\\ x_{2}\left(t\right) \end{array}\right]$, $A=\left[\begin{array}{cc} 0 & 1\\ -k/m & -c/m \end{array}\right]$, $B=\left[\begin{array}{c} 0\\ 1/m \end{array}\right]$, and $C=\left[\begin{array}{cc} 1 & 0\\ 0 & 0 \end{array}\right]$.

*m* is the mass of the overall axial movement of the push platform, *c* is the overall damping coefficient of the push platform, and *k* is the overall elastic coefficient of the push platform. From formula (3), it can be concluded that the transfer function of the axial movement of the push device is

(3) $$\begin{array}{c} H\left(s\right)=\frac{m}{{ms}^{2}+cs+k}. \end{array}$$

### 3.3. Simulation Analysis

Taking the axial motion of the interventional robot as an example, the step signal *y* = 1 is used to simulate the expected axial displacement of the main hand catheter during the actual operation of the doctor [15]. Take formula (3), where *m* = 1 kg, *c* = 0.05 N/(m/s), and *k* = 1.5 N/m. After MATLAB simulation, the simulation results shown in Figure 11 are obtained and the results are in BP for comparison control effects.

Figure 11 is the simulation comparison between the BP neural network PID controller and the traditional PID controller. It can be seen from the results that the overshoot of the system is 20% under the traditional PID control and 12% under the BP neural network PID control. Compared with the traditional PID control, the adjustment time and response speed of the BP neural network PID control are greatly improved. In the actual operation process, doctors need to push the intubation process several times to reach the designated lesion, so reducing the adjustment time is helpful. It can shorten the operation time and improve operational efficiency.

## 4. Experiment

Before the experiment, the specific parameters of the experiment are specified. The axial displacement stroke of the system mechanism is set as 300 mm, and the axial displacement verification experiment of the whole system is divided into two parts: pushing and withdrawing, which ensures that the axial displacement pushing and withdrawing speed is 30 mm/s. This can ensure that the verification experiment is carried out under the premise of the same push speed and the same time delay so as to ensure the authenticity and reliability of the results.

First of all, we use the traditional PID controller to perform basic experiments during the manual control operation [16]. In this case, performance characteristics can be obtained by experiments. Then, we continue to use the designed BP neural network PID controller to improve the accuracy of manual operation. The experimental results obtained by the BP neural network PID controller are shown in Figure 12, and a smooth displacement response without the overshoot is obtained. These two controller axial displacement errors are shown in Figure 13.

The traditional PID controller has many steady-state errors, and its synchronous tracking performance is worse than the BP neural network PID controller. However, although the performance of the BP neural network PID controller is good, due to the communication delay in manual operation, it will cause some errors. The input signal of the system is the pull value of the main end console. The axial displacement value of the main end console is calculated by a mathematical equation, and then these values are converted into the input signal of the stepping motor by the DSP control unit.

Figure 12 shows the axial displacement tracking of the BP neural network PID controller. The new algorithm is suitable not only to reduce the steady-state error and overshoot of the system but also to shorten the rise time and improve the accuracy. Better tracking performance can be achieved. The experimental results show that compared with the traditional PID controller, the overshoot of the new controller is significantly reduced, the axial displacement error is improved, and the tracking speed and accuracy are also significantly improved.

Through the error comparison in Figure 13, we can find that the system under the premise of two different control systems will produce a large error in about 10 s. This is because the stroke of the linear guide rail used in the system is a little small. When the push mechanism is about to reach the end, there will be a large error due to mechanical friction. This is an error in the selection process of mechanical equipment, which will be studied in the future. In order to eliminate this effect, a better linear guide will be selected. In addition, in the whole verification experiment process, the error of push and withdraw also has a certain difference because the motion performance will have a certain change when the motor rotates forward and reverses. In future research, we have to improve the design of the mobile platform, reduce the system error of mechanical equipment, and ensure the reliability of the system.

However, for the modeling of the DC motor, we use a physical method to establish the dynamic model of axial displacement movement, but we need to consider the operation needs under different working conditions, which requires the use of a nonlinear method in modeling and system identification. Most mechanical systems used in the industry consist of motion information such as position and speed. These motion information will show nonlinear behavior in some work areas. For the system with two degrees of freedom (rotation and insertion), when the speed and direction of rotation change, nonlinearity will significantly affect the operation of the system. Therefore, we should pay attention to the nonlinear modeling and parameter identification of system dynamics in the future.

## 5. Conclusions

In this paper, a new catheter operating system of the surgical robot is proposed, and a new mechanical structure of force feedback is designed to measure the near-end force during the operation. Surgeons can also sense the force feedback of the system to avoid misoperation [17]. Secondly, the BP neural network PID controller is designed to improve the motion accuracy of the axial displacement in the process of teleoperation. Compared with the traditional PID control method, the BP neural network PID controller has better control quality.

In the manual control process, the maximum error of the BP neural network PID axial tracking is less than 1.5 mm, and the average error is only 0.48 mm, which basically meets the experimental requirements. Although there are some errors in the axial motion due to the time delay of communication, it can also be used in practical operation. The experimental results show that the BP neural network algorithm is applicable and easy to understand [18].

In the future research work, we will redesign the dynamic model of the catheter operating system of the surgical robot to improve the control accuracy of the system, and through the introduction of the optical fiber sensor and magnetic sensor to form a new collision force acquisition unit, we can obtain the accurate information of the internal force (contact force and friction force) and displacement between the surgical catheter and the blood vessel [19].

## Figures and Tables

**Figure 1:** The da Vinci system.

**Figure 2:** Sensei Xi system.

**Figure 3:** Slave end manipulator of the robot conduit control system.

**Figure 4:** Main end manipulator of the robot conduit control system.

**Figure 5:** Communication diagram.

**Figure 6:** Surgeon's console.

**Figure 7:** Slave end console.

**Figure 8:** Artificial neuron model.

**Figure 9:** BP neural network PID control system.

**Figure 10:** Intelligent adjustment output of parameters *K*_p_, *K*_i_, and *K*_d_.

**Figure 11:** Simulation results.

**Figure 12:** Axial displacement of the BP neural network PID controller.

**Figure 13:** Axial displacement errors of the traditional PID controller and BP neural network PID controller.

## Data Availability

The experiment data used to support the findings of this study are available from the corresponding authors upon request.
